The article "Construction of Music Intelligent Creation Model Based on Convolutional Neural Network" was published in 2022. Journal: Comput Intell Neurosci.

# Construction of Music Intelligent Creation Model Based on Convolutional Neural Network

**DOI:** 10.1155/2022/2854066

**Published:** 2022-07-05

**Authors:** Jing Chen

**Affiliations:** Department of Music, Shandong Women's University, Jinan, Shandong 250002, China

## Abstract

The application of machine learning technology to intelligent music creation has become a very important field in music creation. The main current research on music intelligent creation methods uses fixed coding steps in audio data, which lead to weak feature expression ability. Based on convolutional neural network theory, this paper proposes a deep music intelligent creation method. The model uses a convolutional recurrent neural network to generate an effective hash code, first preprocesses the music signal to obtain a Mel spectrogram, and then inputs it into a pretrained CNN to extract from its convolutional layers. The network space details and the semantic information of musical symbols are used to construct the feature map sequence using selection strategy for the feature map of each convolutional layer, so as to solve the problem of high data feature dimension and poor recognition performance. In the simulation process, the Mel cepstral coefficient method (MFCC) was used to extract the features of four different music signals, and the features that could represent each signal were extracted through the convolutional neural network, and the continuous signals were discretized and reduced. The experimental results show that the high-dimensional music data are dimensionally reduced at the data level. After the data are compressed, the correct rate of intelligent creation is as high as 98%, and the characteristic signal distortion rate is reduced to 5% below, effectively improving the algorithm performance and the ability to create music intelligently.

## 1. Introduction

The application of technology to the intelligent creation of speech and the intelligent creation of musical elements has become two very important fields in the intelligent creation of patterns. The intelligent creation of speech has a good development prospect in social production and life; the intelligent creation of musical elements belongs to an important branch of intelligent creation of patterns, and has been successfully applied in the fields of computer vision such as military, medical, and industrial [1–3]. Since the birth of the world, the research on convolutional neural networks has also made great progress. At present, there are hundreds of convolutional neural networks, among which the representative ones are convolutional neural networks, pattern recognition, music element processing, finance, in the fields of voice intelligent creation, and music element intelligent creation [4–6].

The article "Construction of Music Intelligent Creation Model Based on Convolutional Neural Network" was published in 2022. Journal: Comput Intell Neurosci.

The rapid development of online music has provided great convenience for music operations to acquire music. In order to facilitate user selection, online music usually classifies music, and music classification based on the intelligent creation layer is a common classification method [7–9]. At present, the main process of the intelligent creation classification system in the field of music information retrieval is to first manually extract the music features, then train and model the classifier, and finally input the music features into the built model for intelligent creation classification. But now the manual music feature extraction technology has encountered a bottleneck [10–13]. As a new feature extraction technology, deep learning has achieved excellent performance in the fields of music element processing and natural language understanding. Therefore, this paper uses the powerful feature extraction function of deep learning to find music features that are more suitable for intelligent music creation and classification to design different network structures to classify intelligently based on these musical features. Since the same music may generate different intelligent creation layers, it is difficult to generalize the intelligent creation layer of a single tag at this time, and multiple intelligent creation layer tags are needed to more accurately and comprehensively summarize the intelligent creation layer categories of a piece of music. At the same time, the cognition of the music intelligent creation layer is subjective, so it is necessary to provide a personalized music intelligent creation layer classification for each music operation.

To this end, this paper studies the problem of multilabel personalized classification of music based on an intelligent composition layer. This problem mainly includes two subproblems: the acquisition of the ground-truth labels of the music intelligent creation layer and the personalized classification of music. In response to these two problems, this paper first proposes a method for calculating the personalized truth value of the music intelligence creation layer based on network information and music operation tags. The creative layer personalized truth value is calculated; then a method of mapping the music intelligent creative layer truth value to multilabel categories is proposed, and the specific intelligent creative layer category of music is obtained; finally, a deep convolutional neural network and a random K-label set are used for multilabel classification of musical sentiment with the application of PCA in the intelligent creation of handwritten digits. Although classifiers such as convolutional neural network and SVM have good stability and generalization ability, the high dimensionality of image data makes the time complexity of the algorithm very high, and redundant information will also affect the classification of intelligent creation. In this chapter, principal component analysis (PCA) is used to reduce the dimension of the image data, and the 784-dimensional features of each image in the MNSIT database are reduced to N-59 dimensions. The experimental results show that the running time of the SVM model using the PCA method is greatly reduced, and the classification accuracy is also improved.

The article "Construction of Music Intelligent Creation Model Based on Convolutional Neural Network" was published in 2022. Journal: Comput Intell Neurosci.

## 2. Related Work

With the explosive growth of data, in the context of the era of big data, hash learning plays an increasingly important role in the field of information retrieval. As an important direction of machine learning, hash learning can reduce communication and storage overhead and improve learning and retrieval efficiency. On the other hand, deep learning has been widely studied and applied in academia and industry, and has shown better performance than traditional machine learning methods in the fields of speech intelligent creation, natural language processing, and music element intelligent creation. Recently, some deep hash learning methods have been proposed by combining hash learning and deep learning [14–16].

Zgank [17] proposed to realize creation layer based on a two-layer classifier. The first layer uses the bag-of-users model, which is mainly used for training the general intelligent creation layer classification of music; the second layer uses residual, the model is mainly trained to predict the intelligent creative layer cognition. Anantrasirichai and Bull [18] believes that the two-layer classification method is superior to the traditional one-layer classification method because the method treats the music content itself and specific individual music operations separately. Solanki and Pandey [19] proposed a method based on active learning to realize the personalized classification of the music intelligent creation layer. The method first labels the music data set, and then invites the experimenter to listen to the music on the web page. We can think of this method as an explicit feedback method based on music manipulation. One of the key problems of personalization is the burden of music operation. In order to realize the personalization of different individuals, the participation of music operation is inevitably required to ensure the effect of personalization, but too much participation is also a burden to music operation. Chemical technology has a trade-off in both aspects. Buehler [20] believes that in the aspect of personalization of the music intelligent creation layer, in order to reduce the participation of music operation, it is appropriate to design less music and music operation interaction.

The article "Construction of Music Intelligent Creation Model Based on Convolutional Neural Network" was published in 2022. Journal: Comput Intell Neurosci.

The processing of the true value of the data is different. It first needs to group all music operations according to individual information. For example, according to age grouping, and according to cultural background, music operations can be divided into oriental culture like Western Culture Group [21–24]. After being divided into groups, each group is calculated according to the average value of the music operation labels of all members in the group. Therefore, for personalized music classification based on network information, the burden on music operation is almost zero [25–27].

## 3. Music Grading Based on Convolutional Neural Network

### 3.1. Convolutional Neural Network Hierarchy Division

The layers in the convolutional neural network sort each element of the vector according to the value of *e*, (0 ≤ *i* ≤ *n* − 1) from large to small to obtain a new (creation layer truth value, subscript vector), and select the *k* with the most significant weight elements, the corresponding category can be calculated through the subscript values of these *k* elements, and finally the final category of the song can be calculated for “Music Operation.” The time complexity of the algorithm mainly depends on the sorting time. The complexity is *O*(*n*log*n*), where *i* is the number of classification labels.

First of all, it is necessary to collect the music operation network relationship set:

(1) $$\begin{array}{c} y\left(x,k\right)=\left\{\begin{array}{c} \sum x\left(k,k-1\right)\exp\left(nt\right),\\ \sum x-\exp\left(-\frac{2pi}{nt}\right). \end{array}\right. \end{array}$$

For example, in the network diagram, starting from the nodes in Figure 1, which nodes can be reached by moving a step to the adjacent nodes, that is, which music operations the music operation *uf* pays attention to; starting from the *uf* node, which nodes can be reached by moving two steps to the adjacent node, which can be regarded as the indirect attention to music operation of the music operation *U*, and so on to calculate the distance to other music operations. And it is also necessary to collect the intelligent creation layer classification labels of itself and other music operations for all songs, which are represented by the music intelligent creation layer label vector label set:

(2) $$\begin{array}{c} \frac{s\left(m,n\right)\exp\left(-it/nt\right)}{1-\exp\left(-it/nt\right)}-\frac{\left(m-1\right)\exp\left(-i-t/nt\right)}{1+\exp\left(-it/nt\right)}-1=0. \end{array}$$

We represent the network relationship between music operations by a directed edge with an edge weight of 1 in graph theory. We regard music operations as points of a directed graph. When music operations *uf* pay attention to music operations *uf*, we can use it. In the *F* layer, first arrange each feature map obtained by the S4 layer into a column vector, each feature map has 13 × 13 = 169 features, and then connect all the column vectors in turn, and the final number of features obtained is 169 × 10 = 1690. The extracted features are input into the SVM classifier to obtain the final classification result.

The article "Construction of Music Intelligent Creation Model Based on Convolutional Neural Network" was published in 2022. Journal: Comput Intell Neurosci.

### 3.2. Network Dimensionality Reduction Processing

The number of convolutional layers and the size of the convolution kernel of the first convolutional layer, and the hyperparameters related to dimensionality reduction processing: learning rate, and achieve satisfactory classification performance. It must be carefully adjusted before. In the experiments in this chapter, the set hyperparameters are used without data augmentation:

(3) $$\begin{array}{c} \left\{\begin{array}{cc} 1-k, & 0<k<f\left(k\right)-1,\\ 0, & f\left(k\right)-1<k<f\left(k\right)+1. \end{array}\right. \end{array}$$

The intelligent creation rate of GTZAN dataset is around 73.6%. Given more detailed information on musical style classification, in the form of a confusion matrix, where the columns correspond to the actual styles, the rows correspond to the predicted categories, and the percentage of correct classifications is located on the diagonal of the matrix. Due to the unclear boundaries between some music styles, misjudgment is easy to occur. For example, some classical music has a strong rhythm and is easily mistaken for iazz music; and lock music is easily mistaken for other styles due to its wide range of characteristics, so its classification accuracy is lower than other styles.

Since CNN have many parameters to learn, they cannot be trained efficiently unless there are enough training music elements as shown in Figure 2, so data augmentation has become important to generate more samples of music elements and should list various differences to gain robustness:

(4) $$\begin{array}{c} \sum \frac{x\left(k,k-1\right)}{1-\exp\left(-2\left(pi/nt\right)\right)}-k\frac{\sum x\left(k\right)\exp\left(-2\left(pi/nt\right)\right)}{\exp\left(n\right)-x\left(n\right)}=0. \end{array}$$

However, the experimental results of this chapter are too low to make a very reliable judgment. After further research, it is found that the variation of music repertoire is very rich, so it is not enough to use 100 tracks to represent various variations of a particular genre, and compared with the eight-layer network structure, the training data in this article are too small, so that the final classification result is not particularly ideal. It can be foreseen that with the increase of music repertoire, the intelligent creation effect of this chapter will be further improved.

The article "Construction of Music Intelligent Creation Model Based on Convolutional Neural Network" was published in 2022. Journal: Comput Intell Neurosci.

### 3.3. Principal Component Analysis of Music

The first type of music principal component analysis is to increase the training sample. We extract random 224 × 224 small pieces of music elements from the 256 × 256 music elements. The extracted music elements differ from the original music elements by 32 pixels, so the main part should contain in the training set. The first-Toe method is to use PCA to enhance the training data: a PCA transformation is performed for each RGB music element to complete the denoising function:

(5) $$\begin{array}{c} \frac{k\left(m,n\right)-1}{k\left(m,n\right)+1}-\sum x\left(k\right)-\frac{k\left(m,n\right)}{k\left(m\right)k\left(n\right)-1}=1. \end{array}$$

In the *S* layer, the pooling methods usually selected are average pooling and max pooling, and the average pooling is selected in this chapter. After passing through the S layers, the resulting matrix row and column scales are half the size of the previous layer. It shows that the features of time series and frequency series are manually extracted and put into CNN network training in different combinations, and finally different effects will be obtained. Among them, the intelligent creation rate obtained when all three feature maps are input into the network is the highest, indicating that better results can be obtained only when the training features of Figure 3 are more comprehensive.

To sample the maximum frequency that can be sensed is 20,000 Hz, you need at least 40,000 sampling points per second. The usual sampling rate for real audio files is 44,100 per second, slightly more than 40,000, so we have to consider the same problem when we compress and use at least 40,000 units for input. After obtaining the emotional truth value, for each song's initial value of the truth value is zero vector, this paper proposes a novel method to map the truth value to the specific value. The weighted voting proposed in this paper is different from ordinary voting. It mainly assigns certain weights to the votes of different users according to the node distance in the social network. In the process of accumulating the weights of all votes, different weights value voting has different effects on musical emotion:

(6) $$\begin{array}{c} \sum \frac{x\left(k\right)}{\ln\;k}-\sqrt{x\left(k\right)}-\frac{\left|k\left(m,n\right)\right|}{\left|k\left(m\right)-1\right|}=1. \end{array}$$

The quantitative results of MAE and MSE on the Part A dataset are compared with several algorithms that perform well in this field. As can be seen from the above table, in terms of MSE, the stability error of the algorithm proposed in this chapter is much smaller than that of other algorithms, and the error is reduced by an average of 2.08% compared with the benchmark MCNN. In addition, for the MAE indicator, its algorithm estimation accuracy error is close to MCNN, the best performing algorithm for this indicator.

The article "Construction of Music Intelligent Creation Model Based on Convolutional Neural Network" was published in 2022. Journal: Comput Intell Neurosci.

### 3.4. Network Convolution and Nesting

First, the spectral network convolution graph of each music track is generated, and the time and frequency features of the music track are extracted using the HPSS algorithm. The spectrograms are input to the CNN network together; by adjusting the network parameters, the final intelligent creation result is obtained after training and testing:

(7) $$\begin{array}{c} \sum h\left(k,t-k+1\right)+\sum_{k}h\left(k,t-2\right)=k\sum h\left(k,t-1\right)+\cdots +h\left(k,1\right)+1. \end{array}$$

Usually dropout and momentum can improve learning. Since it takes a long time for the network to converge using dropout for all layers, in the experiments of this chapter.

Figure 4 contains two convolutional layers (layer *C*), two pooling layers (layer *S*), a fully connected layer (layer *F*) and an output layer. In the *C* layer, the size of the convolution kernel is set to 5 × 5, the number of convolution kernels is 5 and 10, and the window-moving step is 1. In the *S* layer, the pooling methods usually selected are average pooling and maximum pooling, and the average pooling is selected in this chapter:

(8) $$\begin{array}{c} \left|\frac{m\left(x,t-y+1\right)-m\left(x,t-1\right)}{f\left(x,t-y+1\right)-f\left(x,t-1\right)}\right|+\left|\frac{m\left(x,1\right)-m\left(x,t-1\right)}{f\left(x,1\right)-f\left(x,t-1\right)}\right|>1. \end{array}$$

The null hypothesis and alternative hypothesis of digital information data are as follows: assuming *t* = 0, if the ADF test value is greater than or equal to the critical value at a certain confidence level, the original hypothesis wind is accepted: *Y* = 0, indicating that the sequence has a unit root and is nonstationary. If the ADF test value is less than the critical value at a certain confidence level, the null hypothesis date is rejected, indicating that the sequence has no unit root and is stable. However, music emotion itself is subjective, and it is based on various influences, so even if the classification accuracy of the trained emotion classifier reaches 100%, it is only based on the average emotion cognition of the public. For different individuals, the classification accuracy is not necessarily the best.

The article "Construction of Music Intelligent Creation Model Based on Convolutional Neural Network" was published in 2022. Journal: Comput Intell Neurosci.

## 4. Construction of an Intelligent Music Creation Model Based on Convolutional Neural Network

### 4.1. Convolutional Neural Network Feature Extraction

A total of 20,000 iterations are performed on the network convolution training samples, when the learning rate is relatively small, the learning process will be very slow, and the intelligent creation rate is still unstable. Appropriate improvement can effectively improve lack of efficiency. In the paper, we found some image data with large estimation error according to the order of group ID. We found that the model performed poorly in some cases where the scene was too dense or the background was too complex. For this reason, we made curve statistics on the population distribution of data sets *A* and *B*. In order to find the imbalanced distribution of the data set itself, the training set rarely contains these complex scenes for learning, resulting in a large error in the estimation of a few extremely dense scenes in the test set. In addition, the scene migration ability of the model needs to be further explored:

(9) $$\begin{array}{c} 1<f\left(m,n\right)<\sqrt{x\left(k\right)}-\sqrt{x\left(k\right)-1}-\sqrt{x\left(k\right)-2}<f\left(m,n\right)-1. \end{array}$$

The stationarity test of time series means that the statistical law of time series does not change with the passage of time, that is, the characteristics of the random process that generates variable time series data do not change with the change of time. Most of the economic variable data involved in economic analysis are time series data, and most of the economic time series are nonstationary, so it is necessary to test the stationarity of the observed time series data.

A total of 50 training rounds, batch size is 25, initial learning rate is 0.8, convolution kernel size is 25, maximum channel number is 128, cavity coefficient is 1, step size is 1, the number of units used by the recurrent neural network is 128, the size of convolution kernel connected between residual networks is 9, loss weight is 0.1 and 2.5*E* − 4. The emotion truth value involved in the emotion-based multilabel personalized classification in this paper is inherently subjective, and it is almost impossible to reach consensus among all cognitive viewpoints in terms of emotion cognition, so it belongs to the second type of truth value. This section mainly discusses the truth value of music emotion involved in this paper. Experimental results show that the proposed CRNNH can achieve superior performance compared to other advanced hashing methods (Figure 5).

### 4.2. Algorithm Training for Intelligent Music Creation

This model is used when the number of categories of music intelligent creation data is greater than two categories. For example, in music classification, music signals are classified into one of folk songs, guzheng, rock, and pop; in Section 4, the classification of handwritten digital intelligent creation, the data labels are 10; in document classification, the model data can be grouped into one of several categories such as sports, economics, entertainment, technology, and more:

(10) $$\begin{array}{c} \overset{f,g<1}{\overset{︷}{f\left(m,n\right)-f\left(m-1,n-1\right),g\left(m,n\right)-g\left(m-1,n-1\right)}}⟶\left[F\left(m,n\right),G\left(m,n\right)\right]. \end{array}$$

According to the music retrieval method based on example semantics, use the improved model to learn the semantic vector of music, use the semantic vector to compare the similarity with the marked data set in the database, and return the similarity in the semantic space according to the cosine similarity calculation method. music. In the experiment, the music in the test set is obtained by the convolution model to obtain the semantic vector, and then the return value is obtained in the labeled corpus. If the labeling accuracy of the algorithm is high, the original songs manually labeled in the corpus can be returned after retrieval. Therefore, set the *K* value in Figure 6, and find the percentage of the first K values that can be returned to the original song.

The article "Construction of Music Intelligent Creation Model Based on Convolutional Neural Network" was published in 2022. Journal: Comput Intell Neurosci.

First of all, we can see that the two tags of regional wind and rock do not belong to the intelligent creation layer tags selected in this paper, so they are directly discarded, so the processed tags are (moved, quiet) and (passion, joy), respectively. Assuming that the music *m*0, *m*1, *m*2 belong to albumo, and *m*3, *m*4, *m*5 belong to albuml, we pass the intelligent creation layer of the playlist to the music in the playlist, then the intelligent creation layer label of *m*0, *m*1, *m*2 is (moved, quiet), while the smart creation layers for *m*3, *m*4, and *m*5 are labeled (passion, joy):

(11) $$\begin{array}{c} \left\{\begin{array}{c} \text{Dertimerst}\left(k,k-1\right)-\text{Dertimerst}\left(1,1\right)\in K\left(0,1\right),\\ \text{hermerts}\left(k\right)-k\in K\left(1,1\right). \end{array}\right. \end{array}$$

For the convenience of discussion, we may assume that the subscript sequence of the intelligent creation layer in this example is moving, loneliness, quiet, warmth, romance, healing, sadness, missing, passion, joy, lovelorn, and nostalgia. So *m*, *m*1, *m*2 smart authoring layer labels can be represented by vectors as (1, 0, 1, 0, 0, 0, 0, 0, 0, 0, 0, 0), *m*3, *m*4, *m*5 smart authoring layer labels can be represented by a vector as (0, 0, 0, 0, 0, 0, 0, 0, 1, 1, 0, 0).

The article "Construction of Music Intelligent Creation Model Based on Convolutional Neural Network" was published in 2022. Journal: Comput Intell Neurosci.

### 4.3. Optimization of the Authoring Model Structure

The larger the number of participants in the experiment, the easier it is to collect more data, but the problem is that it is more difficult to achieve a consistent perception of many musical emotions. When it is difficult for the same music to achieve the same emotional perception among different users, these methods usually average the classification labels. That is, the loss is calculated at each stage of the network, so as to ensure the normal parameter update in network training and solve the problem that the over-deep network is difficult to optimize. By analyzing and comparing a large number of experimental results, it is found that the MSE index of the proposed algorithm is reduced by 2.08% on average compared with the benchmark on the Part A data set for Table 1, so this pretrained convolutional network is used to extract convolutional feature maps.

In this algorithm, each node is visited at least once. If the effective attention relationship is defined as the attention relationship in which the followed user exists in the user set we selected. Then, each effective attention relationship algorithm will only be visited once, so its time complexity depends on the number of nodes in the directed graph and the number of effective attention, so the time complexity of the entire algorithm is: *O*(*m*), the algorithm will only visit once, so its time complexity depends on the number of nodes in the directed graph and the number of effective attention, so the time complexity of the entire algorithm is: O(max(IEI, IUl)), where IEI is the number of effective attention for music operations, IUI is the size of the music operation set we have chosen:

(12) $$\begin{array}{c} \forall w\left(i,j\right)=1,\exists w\left(i\right)+w\left(j\right)+h\left(1-h\right)*w\left(i-1,j-1\right)+h=1. \end{array}$$

First normalize, the classification effect is the best. Each sample in the dataset is 28*∗*28 in size, that is, 784-dimensional data, which means that each sample has 784-dimensional data, which not only increases the training time of the sample but also affects the processing performance of the classifier. That is, the variables are nonstationary, but a certain linear combination of them may be stationary, that is, a group of variables maintain a trend of a group of linear relations within a certain period of time, there is a cointegration relationship between the variables, regression is also useful, a certain linear combination of nonstationary variables can correctly reflect the long-term relationship between them.

The article "Construction of Music Intelligent Creation Model Based on Convolutional Neural Network" was published in 2022. Journal: Comput Intell Neurosci.

## 5. Application and Analysis of Music Intelligent Creation Model Based on Convolutional Neural Network

### 5.1. Convolutional Neural Network Data Pooling

In the intelligent creation classification of convolutional neural network, but when users actually use, only for decoding operation, longer but can obtain better compression effect, can retain encoder part accordingly, and calculation of compression always borne by the service side, although the circulation of the neural network parallel efficiency is quite short, but the decoder does not include circulation part of the neural network, can avoid the high complexity of the neural network. The value of the learning rate 77 is usually in [0, 1]. Learning rate 77 is too large or too small will affect the performance of the network:

(13) $$\begin{array}{c} o\left(k,k-1\right)=\left\{\begin{array}{c} \sum h\left(k\right)w\left(i,k\right)⟶o\left(k\right),\\ \sum a*h\left(k\right)-b*w\left(i,k\right)⟶o\left(k-1\right). \end{array}\right. \end{array}$$

The variable learning rate means that the learning rate is relatively large in the early stage of network training, and as the training process progresses, the learning rate decreases continuously, so that the network in Figure 7 tends to be stable.

The load of these two growth cofactors is below 0.5, but the other factors are above 0.5, indicating that the other variables have high validity. In terms of the price of digital lamination or services, the average score is 3.76, and the standard deviation is 0.73, which is above the middle level. Therefore, the corresponding model compression can only be carried out on the decoding end part.

### 5.2. Realization of Music Intelligent Creation Simulation

Users cannot directly attach emotional labels to music, but can only create a playlist, add a series of music to the playlist, and then attach emotional labels to the playlist, indicates which categories the songs in the playlist are classified into for the user who created the playlist. Since the labels attached by users to the playlist are not limited to emotional category labels, we need to filter the labels, and directly discard the labels that do not belong to the classification category we defined. Therefore, this paper adopts an improved algorithm to optimize the *C* and *g* parameters in SVM, and proposes a support vector machine optimization based on the improved music element group algorithm, the algorithm steps are as follows: (1) Input the training samples with features extracted by the Mel cepstral coefficient method; (2) Initialize the penalty factor *c* and kernel function parameter *g* of the SVM; (3) Initialize the position and velocity of the population, use the accuracy rate obtained by SVM as the fitness function of the PSO algorithm; (4) Update the music element and calculate the fitness function value of the updated music element. At this time, the penalty factor *c* and the kernel function parameter *g* are, respectively, are 73.829 and 0.71441:

(14) $$\begin{array}{c} o\left(x,y\right)-\frac{1-\exp\left(x+y\right)}{1-\exp\left(x\right)*\;\exp\left(y\right)}-\frac{1-\exp\left(x+y\right)}{1+\exp\left(x+y\right)}\overset{x-y<1}{⟶}1-\exp\left(\sqrt{x+y}\right). \end{array}$$

Given a piece of music element it, and the size and number of feature maps of a sample after passing through the layer are different, so the model intelligently composes multiple tags of different musical clips from the MagnaTagATune dataset, which have different styles, moods, and other information about the music. The purpose of this model is to correctly and intelligently create the labels of music files, and randomly scramble the dataset used for experiments. The model in Figure 8 was trained for over 60,000 iterations and completed 100 epochs.

The article "Construction of Music Intelligent Creation Model Based on Convolutional Neural Network" was published in 2022. Journal: Comput Intell Neurosci.

Using regularization matrix three to control the quantization error. Another advantage of three-1 regularization is that compared with L2 regularization, it requires less computational cost and has sparseness, that is, its training process can be smoothly accelerated, and more hash bits are 1 or 0.1, can generate more efficient hash codes. However, optimizing the three-1 regularization term may cause the binary code to be composed of 1s, which will affect the final performance. This is because the optimization of the regularization will affect the balance of the hash code. In order to maintain the balance of the hash code, the square sum balance criterion of the mean value of the hash code is used, and the balance criterion can make the hash code every bit is as consistent as possible a 1 or 0.

### 5.3. Example Application and Analysis

The weighted music operation proposed in this paper is different from the ordinary music operation. It mainly assigns certain weights to the music operations of different music operations according to the distance of the nodes in the network. Therefore, we can usually think that in the image space, the local pixels are relatively closely related, while the distant pixels are weakly related. With local awareness, training parameters can be minimized by simply computing the relationship between each element of the input data and its local neighbors.

For music operation, the music in the training set of it (may be set to mf), we set the true value of the intelligent creation layer of the music operation to the music mf as the true value of the music intelligent creation layer of the training set, which needs to be calculated and obtained by the method proposed in this article, which is also the main work of the personalization of the music intelligent creation layer, see for details; for the music in the music operation *ui* test set (may be set as *mk*), we set the music operation to the music *mk*'s true value of the intelligent creation layer as the training set music intelligence in the truth value of the creation layer, which can be obtained directly through the smart creation layer tag of the music operation. In this paper, unless otherwise specified, all the true values of the music intelligent creation layer mentioned in Table 2 refer to the true values of the training set music intelligent creation layer.

The article "Construction of Music Intelligent Creation Model Based on Convolutional Neural Network" was published in 2022. Journal: Comput Intell Neurosci.

The size of its coefficient represents the size of reliability. When the Cronbach coefficient is above 0.6, the reliability is acceptable. When the Cronbach coefficient is below 0.6, the reliability is insufficient, only average classification accuracy of the convolutional neural network using the variable rate in Figure 9 also reached 92.6% and 91.2%, which are also higher than 90.20% of the traditional convolutional neural network.

This experiment investigates the impact of layers, so the feature map sequence contains {40, 80, 120, 160, 240, 320} feature maps, the smart creation results of different numbers of feature maps are shown in the figure, it can be seen that when bow is set to 24, CRNNH can obtain better smart creation accuracy. The intelligent creation results of feature maps of different sizes are shown in the figure. Better intelligent creation results can be obtained when the image size is 6*∗*6. The two features greatly reduce the training parameters of the neural network; at the same time, they also benefit from the powerful feature abstraction ability of the convolutional neural network. Similarly, music also has some characteristics of images, such as local perception, so this paper also combines it with the powerful feature abstraction ability of convolutional neural network to perform multi-label emotion classification for music, the first is good robustness to imbalanced datasets, and the second is a simple serve as metrics for the entire dataset description in Figure 10.

The experiment uses MAP (mean average precision) and AUC (the area under the receiver operating characteristic curve) as evaluation indicators. MAP finds the average correct rate for each point in the ranking for each retrieved song. The training process of CNN is described in detail, and the performance of the network under different sizes of convolution kernels is compared, and the size of the convolution kernel that can achieve the best network performance is screened. The ROC curve reflects the change in the probability of a positive case being classified as a positive case and the probability of a negative case being mistakenly classified as a positive case. The value of AUC is the size of the area below the ROC curve. Usually, the value of AUC is between 5 and 10, a larger AUC represents better retrieval performance is to return a sorted list according to the decision value for each label in the dataset, and average the retrieval results of all labels. The learning result of the convolutional neural network is performed, and CNN-ELM is the result of the data set being adjusted by the SMOTE algorithm and then classified by the ELM network. CNN-ELM obtains higher accuracy and *F* value, while CNN-SMOTE has higher recall, so the retrieval results will be better than other algorithms. It can be seen that CNN-SMOTE returns seven songs that match the label search terms, which are better than the results before adjustment.

The article "Construction of Music Intelligent Creation Model Based on Convolutional Neural Network" was published in 2022. Journal: Comput Intell Neurosci.

## 6. Conclusion

In order to accurately describe the ability of intelligent music creation, this paper uses the convolutional neural network segmentation algorithm to obtain the pitch frequency of each intelligently created note. A melody representation model was established for the music data set to be retrieved and the input music samples, a genetic algorithm was designed to establish an approximation template for intelligently created music, and the individual differences in the input of intelligently created music were corrected, thereby improving the retrieval accuracy. In order to speed up the retrieval speed, a local hash-sensitive algorithm for intelligent creation retrieval is designed, and an index is established for the music database. The label data of the music intelligent creation layer collected from the online music platform is represented by a vector. For a specific music operation, the true value of each music is calculated by the weight accumulation method of the label data of other music operations. In order to overcome the “semantic gap” problem, the music is mapped to a semantic space, the convolutional neural network model is used to obtain the music semantic features, and the semantic annotation vector is generated for the music according to the semantic features. Replace the Softmax classifier in CNN with the SVM classifier, and compare it with the classic CNN and other related literature. Experiments show that the model can still obtain better labeling results when there are few manually labeled music in the dataset and the labeling samples are unevenly distributed, and can achieve the goal of retrieval in the semantic vector space, and obtain a higher score.

The article "Construction of Music Intelligent Creation Model Based on Convolutional Neural Network" was published in 2022. Journal: Comput Intell Neurosci.

## Figures and Tables

**Figure 1:** Convolutional neural network hierarchical relationship set.

**Figure 2:** Dimensionality reduction processing of convolution kernel network in convolution layer.

**Figure 3:** Music principal component scale factor analysis.

**Figure 4:** Network convolution pooling topology.

**Figure 5:** Convolutional neural network feature extraction spectral distribution.

**Figure 6:** Label distribution of intelligent authoring layer of convolutional neural network.

**Figure 7:** Network data pooling input pretrained network.

**Figure 8:** Sparsity distribution of intelligent music creation.

**Figure 9:** Convolutional neural network weight music operation.

**Figure 10:** Mean square error result of intelligent music creation.

**Table 1:** Authoring model structure optimization algorithm.

Authoring model text	Optimization algorithm steps
*w*(*i*)+*w*(*j*) in the input layer	Import matplotlib.pyplot as plt
Between each *h*(1 − *h*) layer	Import numpy as np
The number of nodes	Import matplotlib as mpl
Excitation function $\sqrt{x\left(k\right)}$	Import settings
Initialize the connection weights	*g*(*m*, *n*) of the hidden layer
Determine the rate and *f*(*m*, *n*)	*X* = np.arange (1, st.tot_det-1, st.step)
Initialize the thresholds *w*(*i*, *j*)	*Y* = np.arange (1, st.tot_det-1, st.step)
1 − exp(*x*+*y*)	Hidden layer and input layer
Calculate the *k*(*m*) − 1 hidden layer	∑*h*(*k*)*w*(*i*, *k*) − *a∗h*(*k*) − *b∗w*(*i*, *k*)⟶*t*
Dertimerst(*c*, *c* − 1) ∈ [0,1,2,…, *c* − 1]	Output layer of the network

**Table 2:** Training set music intelligent creation instructions.

Creation layer	Instructions rate 1	Instructions rate 2	Instructions rate 3	Instructions rate 4
10	0.121	0.993	0.322	0.666
20	0.004	0.553	0.346	0.117
30	0.219	0.213	0.638	0.404
40	0.661	0.742	0.559	0.037
50	0.318	0.338	0.295	0.825
60	0.006	0.086	0.412	0.385

## Data Availability

The data used to support the findings of this study are available from the corresponding author upon request.
